The article "LncMAPK6 drives MAPK6 expression and liver TIC self-renewal" was retracted in 2022. Reasons: results that could not be reproduced; duplicated images; signs of a paper mill; original data or images not available.

# LncMAPK6 drives MAPK6 expression and liver TIC self-renewal

**DOI:** 10.1186/s13046-018-0770-y

**Published:** 2018-05-15

**Authors:** Guanqun Huang, Hui Jiang, Yueming He, Ye Lin, Wuzheng Xia, Yuanwei Luo, Min Liang, Boyun Shi, Xinke Zhou, Zhixiang Jian

**Affiliations:** 1 Department of general surgery, The Fifth Affiliated Hospital of Guangzhou Medical University, Guangdong Sheng, China; 2 Department of Abdominal Oncology, The Fifth Affiliated Hospital of Guangzhou Medical University, Guangdong Sheng, China; 3 Department of General Surgery, Guangdong General Hospital, Guangdong Academy of Medical Sciences, Guangdong Sheng, China

**Keywords:** MAPK6, lncMAPK6, Liver TIC, Self-renewal, Tumor targeting

## Abstract

**Background:**

Liver tumor initiating cells (TICs) have self-renewal and differentiate capacities, and largely contribute to tumor initiation, metastasis and drug resistance. MAPK signaling is a critical pathway in many biological processes, while its role in liver TICs hasn’t been explored.

**Methods:**

Online-available dataset was used for unbiased screening. Liver TICs were examined CD133 FACS or oncosphere formation. TIC self-renewal was detected by oncosphere formation and tumor initiation assay. LncRNA function was detected by loss of function or gain of function assays. The molecular mechanism of lncRNA was explored by RNA pulldown, RNA immunoprecipitation, ChIP, western blot and double FISH.

**Results:**

Here, we examined the expression profiles of MAPK components (MAPKs, MAP2Ks, MAP3Ks, MAP4Ks), and found MAPK6 is most highly expressed in liver cancer samples. Moreover, a divergent lncRNA (long noncoding RNA) of MAPK6, termed lncMAPK6 here, is also overexpressed along with liver tumorigenesis. LncMAPK6 promotes liver tumor propagation and TIC self-renewal through MAPK6. LncMAPK6 interacts with and recruits RNA polymerase II to *MAPK6* promoter, and finally activates the transcription of MAPK6. Through MAPK6 transcriptional regulation, lncMAPK6 drives MARK signaling activation. *LncMAPK6*-MAPK6 pathway can be used for liver TIC targeting. Altogether, lncMAPK6 promotes MARK signaling and the self-renewal of liver TICs through MAPK6 expression.

**Conclusion:**

MAPK6 was the most highly expressed MAPK component in liver cancer and liver TICs and lncMAPK6 participated in the transcriptional regulation of MAPK6in cis. This work revealed the importance role of MAPK signaling in liver TIC self-renewal and added a new layer for liver TIC and MAPK6 expression regulation.

## Background

Liver cancer is a serious cancer type all over the world. Liver cancer bulk contains many kinds of cells, including liver tumor initiating cells. Liver tumor initiating cells (TICs), also termed liver cancer stem cells (CSCs), are the origin of liver tumorigenesis, metastasis, drug-resistance and relapse [16]. Liver TICs can self-renewal and differentiate into a new tumor [33, 34]. Recently, several functional assays of liver TICs have been developed, including gradient xenograft formation, sphere formation, side-population, transwell and xenograft [9, 15, 24]. In these assays, sphere formation and gradient xenograft formation were widely-accepted for liver TICs. Some surface markers have been examined to detect and enrich liver TICs, including CD133, CD13, CD24 and CD90 [11, 21, 38]. However, the biology of liver TICs remains elusive.

The article "LncMAPK6 drives MAPK6 expression and liver TIC self-renewal" was retracted in 2022. Reasons: results that could not be reproduced; duplicated images; signs of a paper mill; original data or images not available.

Several transcription factors participate in the self-renewal of liver TIC, including Zic2, c-Myc, Oct4, Sox4 [8, 41]. The well-known modulators of liver TIC self-renewal are Wnt/β-catenin signaling, Notch signaling, Hedgehog and Yap1 signaling pathways [30, 40, 42, 43]. MAPK signaling pathway, one of the most important pathways in signaling transduction and an integration point for multiple biochemical signals, plays a critical role in tumorigenesis, immunology regulation, growth and development [14, 20, 28, 44]. However, the role of MAPK signaling pathway in liver TICs hasn’t been explored. Here we performed a unbiased screening on the expression profile of MAPK components in liver tumorigenesis, and found MAPK6 (mitogen-activated protein kinase 6) was the most highly expressed MAPK component in liver cancer and liver TICs.

MAPK6 is a member of the Ser/Thr protein kinase family and also termed as Erk3. MAPK6 is related to Arrhythmogenic right ventricular cardiomyopathy (ARVC) and p70S6K Signaling, and associates with pulmonary immaturity [3, 19]. It is known that MARK6 can be phosphorylated at ser-189 and then activate MAPKAPK5, which in turn phosphorylates MARK6 [2]. By similarity, MAPK6 may promote cell cycle entrance. As for tumorigenesis, MARP6 participates in HCC development and non-small-cell lung cancer (NSCLC) development [5, 6]. While, its role in liver TICs is unclear. Here we found MAPK6 is vigorously expressed in liver tumor and TICs. MAPK6 deficient liver TICs showed impaired self-renewal, and MAPK6 overexpression promoted the self-renewal of liver TICs, revealing the critical role of MAPK6 in liver TICs.

Long noncoding RNAs (LncRNAs) are defined as RNA molecules which are longer than 200 nucleotides in length but can’t code protein [4]. Recent studies defined lncRNAs as critical modulators in various physiological and pathological processes, including tumorigenesis [29, 35]. As for tumorigenesis, lncRNAs are involved in tumor formation, colony formation, metastasis, energy metabolism and so on [17, 32, 37, 39]. LncRNAs can combine with chromatin remodeling complexes (SWI/SNF, NURD, NURF, PRC1/2, and so on) and regulate the transcription of target genes [35]. LncRNAs also interact with signaling proteins and change their stability or activity [32, 36]. Here, we found lncMAPK6 and MAPK6 were vigorously expressed in liver TICs. LncMAPK6 and MAPK6 were involved in the maintenance regulation of liver TICs. LncMAPK6 interacted and recruited RNA polymerase II to *MAPK6* promoter to initiate transcription. Moreover, *lncMAPK6*-MAPK6 pathway serve as a target for liver propagation and TIC clearance.

The article "LncMAPK6 drives MAPK6 expression and liver TIC self-renewal" was retracted in 2022. Reasons: results that could not be reproduced; duplicated images; signs of a paper mill; original data or images not available.

## Methods

### Primary samples

The detailed information of these sample was: #1, early HCC, 61 years old, female, tumor size, 7.2 × 6.3 × 5.2 mm, non-metastasis. #4, advanced HCC, 74 years old, male, tumor size, 7.9 × 5.3 × 4.8 mm, metastasis. #5, advanced HCC, 63 years old, female, tumor size, 6.9 × 6.1 × 4.2 mm, non-metastasis.

### Antibodies and reagents

Anti-β-actin antibody and DAPI were purchased from Sigma-Aldrich. Anti-MAPK6 and anti-POLR2A antibodies were from Proteintech. PE-CD133 was obtained from MiltenyiBiotec. T7 RNA polymerase and Biotin RNA Labeling Mix were purchased from Roche. The LightShift Chemiluminescent RNA EMSA and Chemiluminescent Nucleic Acid Detection kits were from Thermo Scientific.

### Oncosphere formation

The oncosphere formation assay was performed as described [40]. Briefly speaking, 5000 HCC cells were cultured in sphere formation medium (N2, B27, 20 ng/ml EGF and 20 ng/ml bFGF, in DMEM/F12) and seeded into Ultra Low Attachment 6-well plates. Two weeks later, oncospheres were counted typical images were taken.

### Tumor propagation and initiating assay

For tumor propagation, 1 × 10^6^ lncMAPK6 silenced, overexpressed or control cells were injected into BALB/c nude mice, which were satisficed 1 month later and tumors were weighted. For tumor-initiation, 10, 1 × 10^2^, 1 × 10^3^, 1 × 10^4^, and 1 × 10^5^ lncMAPK6 silenced cells or overexpressed cells were injected into 6-week-old BALB/c nude mice. The ratios of tumor-free mice and tumor TIC ratios were calculated 3 months later. For each sample, six mice were used for tumor injection.

### Immunohistochemistry

Immunohistochemistry (IHC) was performed as described [41]. For IHC, Tris/EDTA buffer was used for antigen retrieval. The samples were detected by HRP substrates and observed with Nikon-EclipseTi microscopy.

### RNA pulldown

RNA pulldown assay was performed as described [27]. Briefly speaking, biotin-labeled lncMAPK6 transcript was obtained through in vitro transcription, and incubaed in sphere lysate. Streptavidin beads were then added for component enrichment, followed by Western blot or silver staining.

The article "LncMAPK6 drives MAPK6 expression and liver TIC self-renewal" was retracted in 2022. Reasons: results that could not be reproduced; duplicated images; signs of a paper mill; original data or images not available.

### Statistical analysis

For statistical analysis, one-tailed Student’s t tests were used. *P* < 0.05 was defined to be statistically significant. Other than denoted, data were shown as means±s.d. *P < 0.05; **P < 0.01; ***P < 0.001. All experiments were repeated at least three times.

## Results

### MAPK6 was up-regulated in liver tumor and liver TICs

Liver TICs are important for liver tumorigenesis, relapse, metastasis and drug resistance. MAPK signaling pathway is a integration point for multiple biochemical signals. However, the role of MAPK pathway in liver TICs hasn’t been explored. Here we performed a unbiased screening for the expression levels of MAPK components in liver cancers using GSE14520 dataset [23, 26]. Of the MAPK components, MAPK6 is most highly expressed in liver cancer samples (Fig. 1a, b). MAPK6 overexpression levels are related to clinical survival (Fig. 1c). To further examine the high expression of MAPK6 in liver cancer, we detected MAPK6 expression levels with realtime PCR and Western blot. MAPK6 was up-regulated along with liver tumorigenesis (Fig. 1d, e). Of note, MAPK6 expression was also related to cancer severity (Fig. 1d, e).

**Fig. 1:** Overexpression of MAPK6 in liver tumor and TICs. (**a**) Expression profiles of MAPK components were shown as heatmap. Blue denoted low expression and red denoted high expression. (**b**) MAPK6 is highly expressed in liver cancers. (**c**) According to MAPK6 expression, HCC samples were divided into two groups (MAPK6^high^ and MAPK6^low^) for Kaplan–Meier survival analysis. (**d**) MAPK6 expression were examined in 19 peri-tumor samples, 7 early HCC samples (eHCC) and 12 advanced HCC samples (aHCC), and all the results were normalized to the average of peri-tumor expression. (**e**) Immunohistochemistry of MAPK6 in peri-tumor, eHCC and aHCC. Representative images and indicated ratios were shown. (**f**, **g**) MAPK6 mRNA expression in CD133^+^ liver TICs (**f**) or oncospheres (**g**) was examine with realtime PCR. RNA expression levels were normalized to MAPK6 expression in non-TICs. For **b**, data were presented as box and whisker plot, boxes represent interquartile ranges (IQR)

We then examined MAPK6 expression pattern in liver TICs. We isolated liver TICs through surface marker CD133, and found MAPK6 was highly expressed in liver TICs (Fig. 1f). We performed sphere formation assay, and also found high expression of MAPK6 in oncospheres (Fig. 1g).

### High expression of lncMAPK6 in liver cancer and liver TICs

We then explored the regulation mechanism of MAPK6 expression. Firstly, we observed *MAPK6* locus, and found lncRNA ENST00000561318 (hereafter named lncMAPK6) is a divergent lncRNA of MAPK6 (Fig. 2a). Through Northern blot, lncMAPK6 was also highly expressed in HCC samples (Fig. 2b). We then examined lncMAPK6 expression profile through in situ hybridization (ISH). As shown in Fig. 2c, lncMAPK6 was highly expressed in liver cancer.

The article "LncMAPK6 drives MAPK6 expression and liver TIC self-renewal" was retracted in 2022. Reasons: results that could not be reproduced; duplicated images; signs of a paper mill; original data or images not available.

**Fig. 2:** LncMAPK6 is overexpressed in liver tumor and TICs. (**a**) MAPK6 locus was shown. There is a divergent lncRNA (ENST00000561318, termed as lncMAPK6 in this research) in near from MAPK6 locus according to UCSC Genome Browser. (**b**) LncMAPK6 expression levels were detected using Northern blot. 18S rRNA was a loading control. (**c**) 19 peri-tumor, 7 eHCC and 12 aHCC were used for In situ hybridization (ISH). Representative photos and indicated ratios were shown. (**d**) LncMAPK6 expression levels in CD133^+^ liver TICs and CD133^−^ non-TICs were detected by realtime PCR, and non-TIC expression was used for data normalization. (**e**) Spheres and non-spheres were selected, and lncMAPK6 expression was examined with realtime PCR. (**f**, **g**) FISH assay confirmed the high expression of lncMAPK6 in liver TICs (**f**) and oncospheres (**g**). Zic2 and CD133 were markers of liver TICs. Scale bars, C, 50 μm; F, 20 μm

We also detected lncMAPK6 expression in liver TICs. We enriched CD133^+^ liver TICs, examined lncMAPK6 expression with realtime PCR, and found increased lncMAPK6 expression in liver TICs (Fig. 2d). We also performed sphere formation assay and found increased lncMAPK6 expression in oncospheres (Fig. 2e). Fluorescence in situ hybridization (FISH) also confirmed the high expression of lncMAPK6 in liver TICs (Fig. 2f) and oncospheres (Fig. 2g). Altogether, lncMAPK6 was highly expressed in liver tumor and TICs.

### LncMAPK6 activated liver TIC self-renewal

We also detected the role of lncMAPK6 in liver TIC regulation. LncMAPK6 depleted cells were generated for oncosphere formation assay. Sphere formation was inhibited once lncMAPK6 was depleted, indicating the essential role of lncMAPK6 in liver TIC self-renewal (Fig. 3a). We also injected 10, 1 × 10^2^, 1 × 10^3^, 1 × 10^4^ and 1 × 10^5^ lncMAPK6 depleted cells into BALB/c nude mice for tumor initiation, and found impaired tumor initiation (Fig. 3b). The ratios of liver TICs were also decreased upon lncMAPK6 depletion (Fig. 3b). We also found lncMAPK6 was required for the invasion of liver TICs (Fig. 3c). We also silenced lncMAPK6 through antisense oligo (ASO) and performed sphere formation and transwell assays. The results confirmed that lncMAPK6 was required for the self-renewal and invasion of liver TICs (Fig. 3d, e).

The article "LncMAPK6 drives MAPK6 expression and liver TIC self-renewal" was retracted in 2022. Reasons: results that could not be reproduced; duplicated images; signs of a paper mill; original data or images not available.

**Fig. 3:** LncMAPK6 was required for liver TIC self-renewal. (**a**) LncMAPK6 depleted cells were generated through CRISPRi strategy, and sphere formation assay was performed to detect liver TIC self-renewal. LncMAPK6 depletion efficiency was examined by Northern blot (left). Typical photos and the ratios of sphere-initiating cells were shown. (**b**) 10, 1 × 10^2^, 1 × 10^3^, 1 × 10^4^ and 1 × 10^5^ lncMAPK6 depleted cells were used for 3 months’ tumor formation. Tumor initiating cell ratios were analyzed through extreme limiting dilution analysis (right panels). CI, confidence interval. (**c**) Transwell assay was performed using lncMAPK6 silenced cells, and representative images and cell numbers were shown. (**d**, **e**) LncMAPK6 antisense oligo (ASO) treated cells were utilized for sphere formation (**d**) and invasion assay (**e**), and the typical images were shown. (**f**) LncMAPK6 overexpressed cells were established by CRISPRa strategy, and enhanced sphere formation capacity was found in lncMAPK6 overexpressing cells. (**g**) 10, 1 × 10^2^, 1 × 10^3^, 1 × 10^4^ and 1 × 10^5^ lncMAPK6 overexpressed cells were used for 3 months’ tumor initiation

To further confirm the role of lncMAPK6 in liver TICs, we then overexpressed lncMAPK6 through CRISPRa strategy, and found lncMAPK6 overexpression promoted the self-renewal of liver TICs (Fig. 3f). Then we injected 10, 1 × 10^2^, 1 × 10^3^, 1 × 10^4^ and 1 × 10^5^ lncMAPK6 overexpressed cells for tumor initiation, and found lncMAPK6 overexpression promoted tumor formation (Fig. 3g). Altogether, lncMAPK6 played a important role in the self-renewal of liver TICs.

### LncMAPK6 drove MAPK6 expression

Many lncRNAs participate in the transcription of nearby genes, thus we detected whether lncMAPK6 drove the expression of MAPK6. We examined MAPK6 expression levels with lncMAPK6 depleted cells and found decreased MAPK6 expression upon lncMAPK6 knockdown (Fig. 4a). Western blot also found that lncMAPK6 depletion largely impaired MAPK6 expression (Fig. 4b). On the contrary, lncMAPK6 overexpression promoted the expression of MAPK6 (Fig. 4c). Altogether, lncMAPK6 drove the expression of MAPK6.

**Fig. 4:** LncMAPK6 drove MAPK6 expression. (**a**) MAPK6 expression in lncMAPK6 depleted cells was detected using three primary samples. (**b**, **c**) LncMAPK6 depleted (**b**) and overexpressed (**c**) cells were used for MAPK6 examined with immunobloting. CRISPRi-lnc, CRISPRi-lncMAPK6; CRISPRa-lnc, CRISPRa- lncMAPK6. β-actin was a loading control. (**d**) MAPK6 knockout cells were established and sphere formation assay was performed. Typical images and indicated ratios were shown in middle and right panels, respectively. (**e**) 10, 1 × 10^2^, 1 × 10^3^, 1 × 10^4^ and 1 × 10^5^ MAPK6 knockout cells were used for tumor formation. (**f**, **g**) LncMAPK6 was silenced (**f**) or overexpressed (**g**) in MAPK6 knockout cells and lncMAPK6 didn’t participate in liver TIC self-renewal upon MAPK6 was deleted. (**h**, **i**) MAPK6 knockout cells were used for lncMAPK6 knockdown (**h**) or overexpression (**i**), followed by transwell assay

Next we detected the role of MAPK6 in liver TICs. MAPK6 knockout cells were constructed and showed impaired sphere formation capacity, indicating that MAPK6 was necessary for liver TIC self-renewal (Fig. 4d). We also performed tumor initiation with gradient MAPK6 knockout cells, and found MAPK6 knockout largely impaired tumor initiation capacity (Fig. 4e). Meanwhile, MAPK6 knockout cells contained decreased ratios of liver TICs (Fig. 4e). Altogether, MAPK6 was essential in liver TIC self-renewal.

The article "LncMAPK6 drives MAPK6 expression and liver TIC self-renewal" was retracted in 2022. Reasons: results that could not be reproduced; duplicated images; signs of a paper mill; original data or images not available.

We also detected the importance of MAPK6 for lncMAPK6 function. We silenced lncMAPK6 expression in MAPK6 knockout cells, followed by sphere formation. Interestingly, lncMAPK6 had no effect on liver TIC self-renewal upon MAPK6 knockout, revealing the critical function of MAPK6 in lncMAPK6 (Fig. 4f). Similarly, we overexpressed lncMAPK6 in MAPK6 knockout cells and found impaired role of lncMAPK6 (Fig. 4g). Beside sphere formation assay, tumor invasion capacity was also examined. LncMAPK6 had no effect on tumor invasion if MAPK6 was knockout, further confirming the importance of MAPK6 in lncMAPK6 signaling (Fig. 4h, i). Altogether, lncMAPK6 drove liver TIC self-renewal by MAPK6.

### LncMAPK6 recruits RNA polymerase II to *MAPK6* promoter

To investigate the molecular mechanisms of lncMAPK6 in MAPK6 expression and subsequent liver TIC self-renewal, RNA pulldown assay was performed. Mass spectrum was used for protein identification and the interaction between lncMAPK6 and POLR2A was found (Fig. 5a), which was also validated by Western blot (Fig. 5b). LncMAPK6 truncates were also constructed for RNA pulldown. The second region of lncMAPK6 (#2) was required for binding with POLR2A (Fig. 5c). EMSA experiment also confirmed the combination of lncMAPK6 and POLR2A (Fig. 5e). We also examined the physiological interaction of POLR2A and lncMAPK6 with RNA immunoprecipitation (Fig. 5e). Double fluorescence in situ hybridization (double-FISH) was also confirmed the co-localization of lncMAPK6 and POLR2A (Fig. 5f).

**Fig. 5:** LncMAPK6 interacted with RNA polymerase II. (**a**) LncMAPK6 was transcribed in vitro for RNA pulldown, and the denoted band in lncMAPK6 sample was identified as POLR2A. (**b**) The binding of lncMAPK6 and POLR2A was examined by Western blot. (**c**) LncMAPK6 truncates were generated (left panels), and incubated with sphere lysates. The interaction between lncMAPK6 truncates and POLR2A was confirmed (right panels). (**d**) RNA EMSA was performed for the combination between lncMAPK6 and POLR2A. The second truncate of lncMAPK6 was used for RNA EMSA. (**e**) Oncospheres derived from clinical samples were used for RNA immunoprecipitation (RIP) assay, and enrichment of lncMAPK6 were detected with realtime PCR. GAPDH was a control. (**f**) The co-localization of lncMAPK6 and POLR2A was confirmed by double FISH assay. Scale bars, 10 μm. (**g**, **h**) LncMAPK6 depleted (**g**) and overexpressed (**h**) cells were crushed for POLR2A ChIP, followed by detection for *MAPK6* promoter enrichment with realtime PCR

POLR2A, a component of RNA polymerase II, plays a fundamental role in transcriptional initiation. Thus we explored the role of lncMAPK6-POLR2A interaction in MAPK6 transcription. We found POLR2A combined with *MAPK6* promoter in liver TICs, while, their binding was diminished upon lncMAPK6 was depleted (Fig. 5g). On the contrary, lncMAPK6 overexpression largely promoted the binding of POLR2A and *MAPK6* promoter (Fig. 5h). Altogether, lncMAPK6 recruited RNA polymerase II to the promoter of MAPK6 to drive its expression.

The article "LncMAPK6 drives MAPK6 expression and liver TIC self-renewal" was retracted in 2022. Reasons: results that could not be reproduced; duplicated images; signs of a paper mill; original data or images not available.

### *LncMAPK6*-MAPK6 served as a target for liver TIC clearance

Finally, we detected the TIC targeting role of lncMAPK6-MAPK6. We examined the tumor propagation capacity of lncMAPK6 depleted cells and lncMAPK6 overexpressed cells, and found lncMAPK6 played an important role in liver tumor propagation (Fig. 6a, b). We also established *MAPK6* promoter deleted cells, followed by tumor propagation. *MAPK6* promoter or MAPK6 knockout cells also showed impaired propagation (Fig. 6c). We performed immunohistochemistry assay, and the results showed impaired expression of MAPK6 in lncMAPK6 knockout or *MAPK6* promoter depleted tumors, validating the role of lncMAPK6 in MAPK6 expression (Fig. 6d). We obtained tumor cells and found lncMAPK6-MAPK6 pathway was required for the proliferation of tumor cells (Fig. 6e). Meanwhile, lncMAPK6-MAPK6 inhibition also induced a decreased numbers of liver TICs, indicating that lncMAPK6-MAPK6 can be used for liver TIC clearance (Fig. 6f). Taken together, lncMAPK6-MAPK6 blockade inhibited the self-renewal and maintenance of liver TICs.

**Fig. 6:** LncMAPK6-MAPK6 pathway can be targeted for liver TIC clearance. (**a**, **b**) 1 × 10^6^ lncMAPK6 silenced (ASO, A) or overexpressed (oeLnc, **b**) were used for 1 month tumor propagation. 6 BALB/c nude mice were used for each sample. (**c**) 1 × 10^6^ indicated cells were used for tumor propagation and tumor weights were examined one month later. (**d**) The indicated tumors were used for MAPK6 immunohistochemistry. (**e**, **f**) The indicated tumors were stained with Ki67 (**e**) and CD133 (**f**) antibodies for FACS detection. Gating strategy and indicated ratios were shown

The article "LncMAPK6 drives MAPK6 expression and liver TIC self-renewal" was retracted in 2022. Reasons: results that could not be reproduced; duplicated images; signs of a paper mill; original data or images not available.

## Discussion

Wnt/β-catenin, Notch and Hedgehog signaling pathways are well-explored pathways in liver TIC self-renewal. All these signaling pathways are finely regulated. Wnt/β-catenin activation is largely modulated by β-catenin stability or activity [7, 10, 22]. Notch activation is regulated by Notch cleavage and nuclear translocation [40]. Here we found MAPK6, a component of MAPK signaling pathway, is involved in the self-renewal of liver TICs. What’s more, MAPK6 is also precisely regulated by lncMAPK6. LncMAPK6 located onto the *MAPK6* promoter and recruited RNA polymerase II to *MAPK6* promoter, which further activate the transcription activation of MAPK6.

LncRNAs play important roles in many biological processes [25]. Here we found a lncRNA drove the self-renewal of liver TICs through MAPK6. Interestingly, lncMAPK6 is a divergent lncRNA of MAPK6. Divergent lncRNAs are transcribed in the opposite direction from nearby genes [12]. Divergent lncRNAs, often modulate their nearby genes in cis, are positively-related to their nearby genes [12]. As a divergent lncRNA of MAPK6, lncMAPK6 was co-expressed with MAPK6 in liver tumor and TICs. LncMAPK6 regulated the expression of MAPK6 through transcriptional activation. There are several lncRNAs involved in MAPK modulation. MALAT1 drove the proliferation and metastasis of gallbladder cancer cells through MAPK signaling [1]. DBH-AS1 and URHC are required for the proliferation and survival of hepatocellular carcinoma by MAPK activation [13, 18]. Here we found lncMAPK6 promoted MAPK6 expression to drive liver TIC self-renewal, revealing the role of MAPK signaling in liver TIC self-renewal and adding a new layer for MAPK6 transcriptional regulation.

As we know, It is impossible that a lncRNA only target one gene. However, we found lncMAPK6 had impaired role upon MAPK6 was deleted, indicating lncMAPK6 exerted its role mainly through MAPK6. We think several reasons can explain this result. 1. Some lncRNAs may locate at particular subcellular position, and the location limited the number of their target genes. 2. lncRNA targeted some other genes, but these genes weren’t required for the self-renewal of liver TICs; 3. Some lncRNAs participated in the transcriptional regulation through lncRNA transcription process but not lncRNAs themself [31]. The process of lncRNA can activate the transcription of their nearby genes. Meanwhile, our results indicated that MAPK6 participated in the self-renewal of liver TICs, but the molecular mechanism of MAPK6 function is still unclear, which need further investigation. Altogether, lncMAPK6 drove the self-renewal of liver TICs through MAPK6 expression. LncMAPK6-MAPK6 pathway can be used for liver TIC targeting.

The article "LncMAPK6 drives MAPK6 expression and liver TIC self-renewal" was retracted in 2022. Reasons: results that could not be reproduced; duplicated images; signs of a paper mill; original data or images not available.

## Conclusion

MAPK6 was the most highly expressed MAPK component in liver cancer and liver TICs and lncMAPK6 participated in the transcriptional regulation of MAPK6in cis. This work revealed the importance role of MAPK signaling in liver TIC self-renewal and added a new layer for liver TIC and MAPK6 expression regulation.
